RETRACTED

# Moringa isothiocyanate complexed with α-cyclodextrin: a new perspective in neuroblastoma treatment

**DOI:** 10.1186/s12906-017-1876-z

**Published:** 2017-07-14

**Authors:** Sabrina Giacoppo, Renato Iori, Patrick Rollin, Placido Bramanti, Emanuela Mazzon

**Affiliations:** 1 IRCCS Centro Neurolesi “Bonino-Pulejo”, Via Provinciale Palermo, Contrada Casazza, 98124 Messina, Italy; 2 Consiglio per la ricerca in agricoltura e l’analisi dell’economia agraria, Centro di ricerca Agricoltura e Ambiente (CREA-AA), Via di Corticella 133, 40128 Bologna, Italy; 3 Université d’Orléans et CNRS, ICOA, UMR 7311, BP 6759, F-45067 Orléans, France

**Keywords:** SH-SY5Y human neuroblastoma cells, Moringa isothiocyanate, α-CD-complexed moringin, Anti-cancer drug

## Abstract

**Background:**

Several lines of evidence suggest the consume of natural products for cancer prevention or treatment. In particular, isothiocyanates (ITCs) exerting anti-cancer properties, have received great interest as potential chemotherapeutic agents.

This study was designed to assess the anti-proliferative activities of a new preparation of *Moringa oleifera*-derived 4-(α-L-rhamnopyranosyloxy)benzyl ITC (moringin) complexed with alpha-cyclodextrin (moringin + α-CD; MAC) on SH-SY5Y human neuroblastoma cells. This new formulation arises in the attempt to overcome the poor solubility and stability of moringin alone in aqueous media.

**Methods:**

SH-SY5Y cells were cultured and exposed to increasing concentrations of MAC (1.0, 2.5 and 5.0 μg). Cell proliferation was examined by MTT and cell count assays. The cytotoxic activity of the MAC complex was assessed by lactate dehydrogenase (LDH) assay and trypan blue exclusion test. In addition, western blotting analyses for the main apoptosis-related proteins were performed.

**Results:**

Treatment of SH-SY5Y cells with the MAC complex reduced cell growth in concentration dependent manner. Specifically, MAC exhibited a potent action in inhibiting the PI3K/Akt/mTOR pathway, whose aberrant activation was found in many types of cancer. MAC was also found to induce the nuclear factor-κB (NF-κB) p65 activation by phosphorylation and its translocation into the nucleus. Moreover, treatment with MAC was able to down-regulate MAPK pathway (results focused on JNK and p38 expression). Finally, MAC was found to trigger apoptotic death pathway (based on expression levels of cleaved-caspase 3, Bax/Bcl-2 balance, p53 and p21).

**Conclusion:**

These findings suggest that use of MAC complex may open novel perspectives to improve the poor prognosis of patients with neuroblastoma.

## Background

Neuroblastoma (NBL) is the third common pediatric malignancy after leukemia and brain tumors [1]. The global annual incidence is about 1–5 new cases per 100,000 children less than one year of age, of which about 30 new cases are estimated in Italy [2]. Specifically, NBL is an extracranial solid tumor that arises from neural crest precursor cells due to genetic alterations affecting the normal developmental program [3]. Although some history cases are described, the majority of NBL cases appears sporadically [4]. To date, therapeutic approaches available for NBL include surgery, radiation therapy, chemotherapy and stem cell transplantation [5, 6]. Despite the improvements recently obtained, the prognosis of patients with metastatic NBL remains poor [7, 8]. Thus, innovative therapeutic strategies to ameliorate the prognosis of NBL patients need to be developed.

RETRACTED

A current trend in the field of pharmacology leads to look at natural compounds as a source of powerful and effective agents to prevent and treat cancer [9–12].

In this context, isothiocyanates (ITCs) released from their glucosinolate precursors have been shown to inhibit different types of cancer including lung, stomach, colon, liver, bladder, mammary glands, prostate and melanoma [13–18].

The ability of ITCs to inhibit carcinogenesis was first recognized more than 30 years ago with α-naphthyl isothiocyanate [19]. Afterwards, numerous evidences have proved the chemopreventive and chemotherapeutic effects of several ITCs, including sulforaphane, benzyl-isothiocyanate, phenethyl-isothiocyanate and allyl-isothiocyanate [20–23]. Over the years, several potential molecular mechanisms of chemoprevention by ITCs have been proposed, such as the induction of phase II cellular detoxification and antioxidant enzymes as well as the induction of cell cycle arrest and apoptosis [24, 25].

The glycosylated compound 4 -(α-L-rhamnopyranosyloxy)benzyl ITC, also known as moringin or GMG-ITC, resulting from myrosinase quantitative hydrolysis under neutral condition (Fig. 1) of glucomoringin (GMG), a GL present in a large quantity in *Moringa oleifera* seeds, was recently characterized [26]. Moringin has been shown to exert an effective antitumor-promoting activity in in vitro and in vivo studies involving a variety of cancer cell lines such as astrocytoma, leukemia and myeloma [27–30]. However, the antitumor effect of moringin against pediatric cancers like human NBL is still unclear.

**Fig. 1:** Production of 4-(α-L-rhamnosyloxy)benzyl isothiocyanate (GMG-ITC; moringin) by myrosinase-catalyzed hydrolysis of glucomoringin (GMG), isolated from *M. oleifera* seeds

Moringin is a solid, odorless, stable compound that can be purified in gram-amounts mainly from seeds of the most widely distributed *Moringa oleifera* Lam. [31, 32] However, like most ITCs, moringin is very poorly soluble in water and unstable in buffered solutions, due to the high electrophilic character of the N = C = S function. Therefore, in order to avoid the use of toxic solubilizers and to overcome the poor solubility of the ITC, we formulated a new complex of moringin with α-cyclodextrin (α-CD; MAC). α-cyclodextrin is a cyclic hexamer of D-glucose that can form water-soluble inclusion complexes with small molecules. Besides, α-CD is Generally Recognized As Safe (GRAS) for use in processed foods at a level of up to 3% (*w*/w) and doses of 10–25 g α-CD were well tolerated by adult human and it is also biocompatible [33, 34]. The formation of a stable MAC complex, with a 1:1 M ratio was initially demonstrated by Roselli et al. [35]. Subsequently, the therapeutic effects of the MAC complex was confirmed by our research group in a recent paper, which examined the anti-inflammatory effects of this new formulation on lipopolysaccharide (LPS)-stimulated RAW 264.7 macrophage cells [36].

RETRACTED

In light of those previous results, the present work aimed to investigate the in vitro anti-proliferative activity of MAC on SH-SY5Y human NBL cell line and to identify the underlying signaling mechanisms resulting in cell death.

## Methods

### Purification of moringin and preparation of MAC complex

Moringin was isolated from *M. oleifera* (fam. Moringaceae) seeds (cake powder PKM2 provided by Indena India Pvt. Ltd.; Bangalore, India) at the Bologna laboratory (CREA-AA; previously CIN) using established methods [26, 28]. Based on the molecular weights and a 1:1 M ratio of the two constituents, a soluble complex was obtained by adding 103 mg of solid moringin to a solution of 300 mg α-CD (Wacker Chemie AG, Germany) in 3.0 mL of water. The resulting aqueous solution was filtered with 0.45 μm filter, then freeze-dried (Edwards model DO1; Milan, Italy). For structural and biochemical studies, three separate preparations of the MAC complex have been performed. Specifically, these preparations were designed to have reproducibility of conjugation between α-CD and ITC through formation of a stable supramolecular structure, to perform structural and biochemical studies and also to have a sufficient amount for all biological evaluations.

### Cell culture conditions and drug treatment

The experiments were carried out on the SH-SY5Y human NBL cell line. SH-SY5Y cells were cultured in monolayer using DMEM medium (Carlo Erba, Italy) supplemented with 10% fetal bovine serum (FBS) (Sigma-Aldrich Co. Ltd., USA). The cells were grown in logarithmic phase at 37 °C in a 95% air/5% CO_2_ humidified incubator. For drug treatment, cells were grown until 70%–80% confluence and incubated for 24, 48 and 72 h (proliferation assays) or for 24 h (for the other assays) with MAC at the following concentration range: 1.0 μg (1.025 nmol/ml), 2.5 μg (2.05 nmol/ml) and 5.0 μg (4.1 nmol/ml).

RETRACTED

### Cell proliferation and cytotoxicity assays

The anti-proliferative activity of MAC was measured by the quantitative colorimetric MTT (thiazolyl blue tetrazolium bromide) assay and cellular counting. SH-SY5Y cells 1 × 10^4^ cells/ml) were seeded into a 96-well culture plate and treated with MAC at different concentrations (1.0, 2.5 and 5.0 μg) for 24, 48 or 72 h. 5-fluorouracil (5-FU) was considered the positive standard. The cell growth was evaluated both spectrophotometrically (Δ absorbance 570-690 nm %) using a microplate reader (Microplate Photometer iMARK™, Biorad). Differences in cell proliferation were estimated as a percentage of growth rates of treated cells compared to untreated ones. Cell growth was also detected by the cell count assay performed by using a Neubauer hemocytometric chamber and counted by an optical microscope (Leica DM 2000 combined with Leica ICC50 HD camera). All experiments were carried out in triplicate and repeated three times.

In addition, possible drug cytotoxicity was assessed by lactate dehydrogenase (LDH) assay and trypan blue dye (0.4% *w*/*v*; TB) exclusion test after 24 h of MAC treatment. LDH concentrations in the medium of treated and untreated cells were measured by a commercial kit (CytiTox 96® Non- Radioactive Cytotoxicity Assay, Promega, Milan, Italy) according to the manufacture’s recommended protocol. The absorbance was quantified spectrophotometrically at 490 nm. LDH levels are extrapolated as the values detected in control cells, which are arbitrarily expressed as 1. The trypan blue dye exclusion assay was used to detect dead cells that were reported as the percentage of stained (non-viable) vs total cells counted. All experiments were performed in triplicate and repeated three times.

### Western blot analysis

For western blot analysis, SH-SY5Y cells were harvested following 24 h of incubation. After washing with ice-cold PBS, the cells were lysed using a buffer consists of 320 mM sucrose, 10 mM Tris-HCl, pH 7.4, 1 mM EGTA, 2 mM EDTA, 5 mM NaN_3_, 50 mM NaF, β-mercaptoethanol, and protease/phosphatase inhibitor mixture (Roche, USA) in ice for 15 min, followed by centrifugation at 1000 g for 10 min at 4 °C. The resulting supernatant was served as cytoplasmic fraction. The pellet was further lysed using a buffer consists of 150 mM NaCl, 10 mM Tris-HCl (pH 7.4), 1 mM EGTA, 1 mM EDTA, Triton X-100, and protease/phosphatase inhibitor mixture (Roche, USA) in ice for 15 min, followed by centrifugation at 15,000 g for 30 min at 4 °C. The resulting supernatant was served as nuclear fraction. Protein concentration was assayed by using the Bradford assay (Bio-Rad, Segrate, Italy). Twenty micrograms of proteins were subjected to sodium dodecyl sulfate-polyacrylamide gel electrophoresis, followed by blotting with PVDF membranes (Immobilon-P Transfer membrane, Millipore). Then, membranes were incubated in blocking solution (5% skimmed milk in 1X phosphate buffered saline) for 45 min at room temperature. After, membranes were incubated with selective primary antibodies for overnight at 4 °C.

RETRACTED

The following primary antibodies were used: phospho-PI3Kinase (1:750 Cell Signaling Technology); PI3Kinase (1:1000; Cell Signaling Technology); phospho-Akt (1:750 Cell Signaling Technology); Akt (1:1000; Cell Signaling Technology); phospho-mTOR (1:750 Cell Signaling Technology); mTOR (1:1000; Cell Signaling Technology); NFkBp65 (1:500, Cell Signaling Technology), IkB-alpha (1:500, Cell Signaling Technology); p-JNK (1:750; Santa Cruz Biotechnology Inc); JNK (1:1000; Santa Cruz Biotechnology Inc); p-p38 (1:750; Cell Signaling Technology), p38 (1:1000; Cell Signaling Technology); cleaved-caspase 3 (1:1000, Cell Signaling Technology) Bax (1:500, Cell Signaling Technology), Bcl-2 (1:500, Cell Signaling Technology), p53 (1:500, Millipore) and p21 (1:1000, Millipore), in 1× PBS, 5% (*w*/*v*) non-fat dried milk, 0.1% Tween-20). Then, membranes were incubated with HRP-conjugated anti-mouse or rabbit IgG secondary antibody (1:2000; Santa Cruz Biotechnology Inc) for 1 h at room temperature. To assess equal loading of proteins, membranes were stripped and reprobed with HRP-conjugated GAPDH (1:1000; Cell Signaling Technology) and Laminin B1 (1:1000 Cell Signaling Technology). Images of protein bands were visualized using an enhanced chemiluminescence system (Luminata Western HRP Substrates, Millipore) and then acquired and quantified with ChemiDoc™ MP System (Bio-Rad) and a computer program (ImageJ software) respectively. The western blot analysis figure is representative of three separate and reproducible experiments.

### Statistical data analysis

Statistical significance of the experimental data was analyzed by one-way ANOVA test, followed by Bonferroni post hoc test for multiple comparisons (GraphPad Software, La Jolla, CA, USA). *p* less than or equal to 0.05 was considered statistically significant. Results are expressed as mean ± SEM.

## Results

### Evidences about MAC capability to interfere with SH-SY5Y cells proliferation

The measurement of cell viability and proliferation was performed to assess the SH-SY5Y cell survival following exposure to increasing concentrations of MAC complex (1.0, 2.5 and 5.0 μg) for 24, 48 or 72 h. At the end of the incubation period, cell proliferation by MTT assay (Fig. 1b) and cell counting were performed (Fig. 2a). MAC treatment was found to reduce cell proliferation in a concentration- and time-dependent manner. In the same conditions, the positive standard, 5-FU showed a greater effect on SH-SY5Y cells than MAC. The MTT data were confirmed by the analysis of the growth curve obtained by counting the cells in a Neubauer hemocytometer chamber after MAC administration for 24, 48 and 72 h (Fig. 2b). In addition, the LDH assay and trypan blue dye exclusion test (cell death) were performed to assess whether the reduction of cell proliferation induced by MAC was due to a cytotoxic effect (Fig. 2c). Our results showed that at concentrations ranging from 1.0 to 5.0 μg, MAC complex did not cause significant increase of LDH release and cell death (Fig. 2d). Moreover, in previous evaluations we evaluated the 10 μg dose, which was found to cause significant SH-SY5Y cell death. Therefore, for all subsequent experimental evaluations, we used concentration of MAC not exceeding 5 μg.

RETRACTED

**Fig. 2:** Anti-proliferative effects of MAC on SH-SY5Y cell line. Cells were cultured in the presence of increased concentrations of MAC for 24, 48 and 72 h. Proliferation rates of SH-SY5Y cells were evaluated by MTT. 5-FU was considered the positive standard (**a**). Results of MTT are expressed as percentage ± SEM of absorbance detected in treated cells. The MTT data were confirmed by the analysis of the growth curve obtained by counting the cells in a Neubauer hemocytometer chamber after MAC administration for 24, 48 and 72 h (**b**). The cytotoxic activities of MAC exposure for 24 h was evaluated in terms of both LDH release (**c**) and cell death (**d**). LDH levels are extrapolated as the values detected in control cells which are arbitrarily expressed as 1. Cell death was reported as the percentage of blue stained (non-viable) vs total cells counted. Data, expressed as mean ± SEM, represent the values obtained in three different sets of experiments made in triplicate. . ^*^ *p* = 0.01 vs CTR; ^**^ *p =* 0.001; ^****^ *p* < 0.0001 vs CTR

### Inhibition of PI3K/Akt/mTOR signaling in response to MAC in SH-SY5Y cells

Recent evidence demonstrates that the activation of the phosphatidylinositol 3-kinase (PI3K)/Akt (protein kinase B)/mammalian target of rapamycin (mTOR) pathway, one of the most potent pro-survival pathway, is involved in NBL progression and correlated also with poor prognosis [37, 38]. Thus, western blot analysis was performed to observe the modulation of the PI3K/Akt/mTOR signaling in SH-SY5Y incubated with MAC for 24 h. Specifically, we focused on the phosphorylation status of PI3K/Akt/mTOR as its activation is mediated by phosphorylation of the proteins involved. Our results showed a significant activation of the PI3K/Akt/mTOR pathway in untreated SH-SY5Y cells, as evidenced by increased expression of p-PI3K (Fig. 3a), p-AKT (Fig. 3b), and p-mTOR (Fig. 3c). Conversely, MAC administration induced a significant downregulation of this pathway.

RETRACTED

**Fig. 3:** Inhibition of PI3K/Akt/mTOR and MAPK pathways in response to MAC in SH-SY5Y cells. Western blot analysis for pPI3K (**a**). CTR vs 1.0 μg ^**^ *p =* 0.0017; CTR vs 2.5 μg ^***^ *p =* 0,0001; CTR vs 5.0 μg ^****^ *p* < 0.0001; 1.0 μg vs 5.0 μg ^*^ *p =* 0,0409. Western blot for pAKT (**b**). CTR vs 5.0 μg ^**^ *p* = 0,0011; 1.0 μg vs 5.0 μg ^**^ *p* = 0,0021; 2.5 μg vs 5.0 μg ^**^ *p =* 0,0019. Western blot for pmTOR (**c**) CTR vs 2.5 μg ^**^ *p =* 0.0017; CTR vs 5.0 μg ^****^ *p* < 0.0001; 1.0 μg vs 2.5 μg ^***^ *p* = 0,0005; 1.0 μg vs 5.0 μg ^****^ *p* < 0.0001; 2.5 μg vs 5.0 μg ^***^ *p =* 0,0002. Western blot analysis for pJNK (**d**). CTR vs 1.0 μg ^***^ *p =* 0.0001; CTR vs 2.5 μg ^****^ *p* < 0.0001; CTR vs 5.0 μg ^****^ *p* < 0.0001; 1.0 μg vs 2.5 μg ^*^ *p =* 0,0122; 1.0 μg vs 5.0 μg ^*^ *p =* 0,0242. Western blot analysis for pp38 (E). CTR vs 1.0 μg ^****^ *p* < 0.0001; CTR vs 2.5 μg ^****^ *p* < 0.0001; CTR vs 5.0 μg ^****^ *p* < 0.0001; 1.0 μg vs 5.0 μg ^****^ *p* < 0.0001; 2.5 μg vs 5.0 μg ^****^ *p* < 0.0001. Results were analyzed by one-way ANOVA followed by a Bonferroni test for multiple comparisons. Blots are representative of three separate and reproducible experiments. The statistical analysis was carried out on three repeated blots performed on separate experiments

### MAC regulates the expression of MAPK pathway in in SH-SY5Y cells

PI3K/Akt/mTOR signaling leads to trigger a variety of intracellular pathways, including the mitogen-activated protein kinase (MAPK) pathway, which plays a pivotal role in regulating many cell functions including survival, proliferation and apoptosis in different cell types [39]. Western blot analysis for c-Jun N-terminal protein kinase (JNK) (Fig. 3d) and p38 (Fig. 3e) revealed that MAPK signaling pathway is intensely activated in SH-SY5Y untreated cells, while MAC administration diminished the expression levels of these markers in a dose-dependent manner.

### Effect of MAC on IκB-α degradation and NF-κB activation in SH-SY5Y cells

Having established that MAC counteracts SH-SY5Y cell proliferation, we have evaluated what are the mediators involved in this process. NF-kB is a dimeric transcription factor normally present in the cytoplasm of cells in an inactive form due to its association with a class of inhibitory proteins called IκBs. Once activated, NF-kB translocates from cytosol to nucleus, where it induces gene expression [40]. Western blot analysis of nuclear fraction indicates that NF-kB expression increased in SH-SY5Y cells treated with MAC when compared to untreated ones, showing a concentration-dependent effect (Fig. 4a). IκB-α degradation is an essential step for NF-kB activation. In parallel, we observed a dose-dependently decrease of cytoplasmic IκB-α expression in SH-SY5Y cells treated with MAC compared to untreated cells. (Fig. 4b). These results suggest that treatment with MAC may play an important role in the regulation of cell viability and NF-kB pathway activation in SH-SY5Y cells.

RETRACTED

**Fig. 4:** Effect of MAC on NF-κB activation and IκB-α degradation and in SH-SY5Y cells. Western blot analysis for NF-κB (**a**). CTR vs 2.5 μg ^****^ *p* < 0.0001; CTR vs 5.0 μg ^****^ *p* < 0.0001; 1.0 μg vs 2.5 μg ^****^ *p* < 0.0001; 1.0 μg vs 5.0 μg ^****^ *p* < 0.0001; 2.5 μg vs 5.0 μg ^*^ *p* = 0,0330.Western blot analysis for IκB-α (**b**). CTR vs 1.0 μg ^****^ *p* < 0.0001; CTR vs 2.5 μg ^****^ *p* < 0.0001; CTR vs 5.0 μg ^****^ *p* < 0.0001; 1.0 μg vs 2.5 μg ^***^ *p* = 0.0006; 1.0 μg vs 5.0 μg ^***^ *p* = 0.0014. Results were analyzed by one-way ANOVA followed by a Bonferroni test for multiple comparisons. Blots are representative of three separate and reproducible experiments. The statistical analysis was carried out on three repeated blots performed on separate experiments

### MAC regulates apoptosis pathway in SH-SY5Y cells

In order to examine the intracellular pathways involved in MAC-induced activation of programmed cell death in SH-SY5Y cells, the expression of main proteins regulating apoptosis, such as cleaved caspase-3, Bax, Bcl-2, p53 and p21 was evaluated by western blot analysis. Apoptosis can be triggered by the activation of caspases, and in particular caspase-3, together with other important key regulators of apoptosis. Western blot analysis performed on SH-SY5Y NBL cell line, showed that treatment of SH-SY5Y with MAC for 24 h caused a significant augmentation of cleaved caspase-3 expression, which was very prominent at 5.0 μg dose (Fig. 5a). Moreover, consistent with the cleavage of caspase, MAC was also able to modulate the Bax/Bcl2 ratio (Fig. 5b and c). In parallel, the expression of proteins in the mitochondrial p53 pathway and one of its target genes, p21, were investigated by western blot analysis. SH-SY5Y cell treated with MAC exhibited a significant increase in p53 (Fig. 5d) and p21 (Fig. 5e) expression levels, when compared to untreated cells. Summarizing, our results revealed that MAC probably induced apoptosis in a dose-dependent manner.

RETRACTED

**Fig. 5:** MAC induces apoptosis pathway in SH-SY5Y cells. Western blot analysis for cleaved caspase-3 (**a**). CTR vs 1.0 μg ^**^ *p* = 0,0056; CTR vs 5.0 μg ^****^ *p* < 0.0001; 1.0 μg vs 2.5 μg ^**^ *p* = 0.0022; 1.0 μg vs 5.0 μg ^****^ *p* < 0.0001; 2.5 μg vs 5.0 μg ^****^ *p* < 0.0001. Western blot analysis for Bax (**b**). CTR vs 5.0 μg ^****^ *p* < 0.0001; 1.0 μg vs 5.0 μg ^****^ *p* < 0.0001; 2.5 μg vs 5.0 μg ^****^ *p* < 0.0001. Western blot analysis for Bcl-2 (**c**). CTR vs 5.0 μg ^****^ *p* < 0.0001; 1.0 μg vs 2.5 μg ^*^ *p* = 0.0006; 1.0 μg vs 5.0 μg ^****^ *p* < 0.0001; 2.5 μg vs 5.0 μg ^****^ *p* < 0.0001. Western blot analysis for p53 (**d**). CTR vs 1.0 μg ^**^ *p* = 0,0032; CTR vs 2.5 μg ^***^ *p* = 0,0001; CTR vs 5.0 μg ^**^ *p* = 0,0092; 1.0 μg vs 5.0 μg ^****^ *p* < 0.0001; 2.5 μg vs 5.0 μg ^****^ *p* < 0.0001. Western blot analysis for p21 (**e**). CTR vs 2.5 μg ^**^ *p* = 0,0129; CTR vs 5.0 μg ^****^ *p* < 0.0001; 1.0 μg vs 2.5 μg ^*^ *p* = 0.0129; 1.0 μg vs 5.0 μg ^****^ *p* < 0.0001; 2.5 μg vs 5.0 μg ^****^ *p* < 0.0001. Results were analyzed by one-way ANOVA followed by a Bonferroni test for multiple comparisons. Blots are representative of three separate and reproducible experiments. The statistical analysis was carried out on three repeated blots performed on separate experiments

## Discussion

To date, there are no definitively effective treatments available for NBL patients. Although, some advances in NBL cure have been obtained in the last years, the therapeutic approaches remain very invasive and the prognosis of NBL patients remains poor [3, 6, 41]. The present study introduces a new application of moringin in the form of the α-cyclodextrin complex (moringin + α-CD; MAC) as a promising therapeutic option in NBL treatment. The complexation of moringin by α-CD results in improving the poor solubility of the ITC through formation of a stable supramolecular structure.

It is well-recognized that a malignant cell transformation and tumor development is characterized by an up-regulated cell number: this is a result of either proliferation or a decreasing in apoptosis [42]. For this reason, many target therapies are focused in counteracting abnormalities of cell cycle. The main goal of successful anticancer drug should be to kill or incapacitate cancer cells without causing excessive damage to normal cells. This ideal condition is possible by inducing apoptosis in cancer cells [43]. This study was designed to verify whether cellular apoptotic induction and cytotoxic properties of the MAC complex causing dose-dependent reduction of viability of human SH-SY5Y cells, a commonly used cell line in NBL studies.

RETRACTED

Interestingly, our observations showed that treatment of SH-SY5Y with MAC caused a significant decrease of cell proliferation in a concentration- and time-dependent manner. Moreover, the growth inhibitory effects of MAC is not mediated by a cytotoxic effect, because at the concentrations used in this experimental study, we did not observe relevant increase in cell death and LDH release. These observations propose MAC as an effective and safe anti-proliferative agent. Our work is consistent with a previous study [44] where synthetic sulforaphane, another widely examined ITC present in cruciferous vegetables, was proved to inhibit cell proliferation by inducing apoptosis in human SH-SY5Y cells. However, we demonstrated the efficacy of MAC at much lower concentrations in comparison with sulforaphane. Therefore MAC complex resulted in a significantly higher efficacy of the active principle than that obtained using the ITC alone.

In addition, in the effort to identify a new therapy that specifically targets the pathways responsible for malignant transformation and progression, we looked at the involvement of the PI3K/Akt/mTOR pathway in NBL progression.

The PI3K/Akt/mTOR signaling indeed seems to be one of the most potent pro-survival pathways involved in NBL tumorigenesis [21, 45]. Specifically, its aberrant activation is common in NBL and also correlates with poor prognosis [37, 46, 47]. Thus, the inhibition of PI3K/Akt/mTOR pathway might prove clinically effective in NBL treatment [47]. To date, there is no data regarding the effects of MAC in the PI3K/Akt/mTOR activity in NBL. Thus, we investigated the role of MAC in modulating the PI3K/Akt/mTOR pathway in SH-SY5Y cells. Western blot analyses showed a significant up-regulation of the PI3K/Akt/mTOR signaling in untreated SH-SY5Y cells, as proven by enhanced phosphorylation of PI3K, Akt and mTOR. On the contrary, a significant dose-dependent decrease of p-PI3K, p-AKT, and p-mTOR was observed in MAC-treated cells.

A recent study suggested that the anti-cancer activity of indole compounds, resulting from hydrolysis of the corresponding glucosinolates and present in large amounts in cruciferous vegetables, could be ascribed to the crosstalk between PI3K/Akt/mTOR signaling and NF-κB pathway [48].

NF-κB regulates cell growth, differentiation and apoptosis by interacting with several upstream and downstream signaling pathways, like PI3K/Akt/mTOR one [48]. mTOR controls Akt via a feedback mechanism, which causes the downstream phosphorylation of IκB-α, and the consequent translocation of NF-κB into the nucleus [48, 49].

RETRACTED

Consistent with these observations, our results showed a significant dose-dependent increase of NF-κB and in parallel a decrease of IκB-α expression levels in MAC-treated cells, compared to untreated ones. Moreover, phosphorylation of the PI3K/Akt/mTOR pathway can lead in turn to triggering a variety of intracellular pathways, like the mitogen-activated protein kinase (MAPK) one [39]. Among the many cell functions in which MAPKs are involved, it has been demonstrated mainly that MAPKs are a pro-survival factor and contribute to the regulation of cell proliferation [50]. Here, in order to investigate whether moringin + α-CD could inhibit MAPKs expression, via PI3K/Akt/mTOR pathway, we looked at the phosphorylation status of JNK and p38 proteins. Our results showed that SH-SY5Y cells treated with MAC exhibited a marked down-regulation in pJNK as well as pp38 expression, suggesting that growth inhibitory activity of MAC is associated with the downregulation of cell proliferation and survival pathway.

Moreover, with a view to confirming that inhibition of survival pathways MAPK lastly leads to SH-SY5Y cell death, we evaluated the expression of main proteins regulating apoptosis. It has been proposed that resistance to extrinsic apoptosis pathway activation is one of the mechanisms that contributes to the aggressive behavior of advanced-stage NBL [51].

Apoptosis is a complex mechanism tightly regulated by several factors. One of the key steps involved in triggering of apoptotic cascade is the leakage of cytochrome C from the mitochondria and subsequent activation of caspases [52]. Several studies reported that phytochemical compounds of *M. oleifera* were able to induce apoptosis in cancer cells [27, 53, 54]. In particular, moringin, the ITC resulting from myrosinase-catalysed hydrolysis of glucomoringin (GMG-ITC) was found to induce caspase 3-dependent apoptosis in multiple myeloma [28]. Here, we showed that SH-SY5Y cells treated with MAC complex exhibited a significant augmentation of cleaved caspase 3 expression, suggesting its involvement in mitochondria-mediated apoptosis. Therefore, we evaluated also the role of MAC in triggering cell death by looking to the main apoptosis-regulatory genes, such as Bax and Bcl-2. In agreement with previous studies reporting the Bax/Bcl-2 modulation and apoptosis-inducing efficacy of ITCs in various human cancer cells [22, 30], we found dose-dependent upregulation of Bax and a downregulation of Bcl-2 in SH-SY5Y cells treated with MAC.

Furthermore, it is estimated that more than 50% of human tumors contain a mutation or deletion of the p53 gene. [55]. Protein p53 is known to play a key role in the mitochondrial intrinsic apoptosis pathway deciding cell fate choices and the activation of several target genes that control apoptosis [56]. Therefore, we believed important to evaluate the ability of MAC to activate p53 and one of its target genes, p21 to induce apoptosis in SH-SY5Y cells. Our results demonstrated a significant expression of p53 as well as of p21 in SH-SY5Y cells incubated with MAC, indicating yet a concentration-dependent effect. Schematically, it is provided a summary figure about the proposal mechanism of action of MAC complex in inducing SH-SY5Y cell death (Fig. 6).

RETRACTED

**Fig. 6:** Summary of MAC complex activity and new therapeutic perspectives. The anti-proliferative action of moringin + α-CD is due to inhibition of the survival PI3K/Akt/mTOR and MAPKs pathways, resulting at last in apoptotic cell death of SH-SY5Y cells

## Conclusion

These findings showed the importance of a new formulation of moringin complexed with α-CD (moringin + α-CD) as a therapeutic target in NBL. Our results revealed that MAC inhibits the proliferation of malignant cell line through activation of apoptosis or programmed cell death in SH-SY5Y cells. In specific, the anti- proliferative efficacy of MAC is ascribed to its ability into inhibiting the survival PI3K/Akt/mTOR and MAPKs pathways, finally resulting in cell death.

## Abbreviations

GMG: glucomoringin
ITCs: isothiocyanates
JNK: c-Jun N-terminal protein kinase
LPS: lipopolysaccharide
MAPK: mitogen-activated protein kinase
MTT: thiazolyl blue
NBL: Neuroblastoma
PI3K/AKT/mTOR: phosphatidylinositol 3-kinase (PI3K)/Akt (protein kinase B)/mammalian target of rapamycin (mTOR)
α-CD: α-cyclodextrin
